# SEMA3B but Not CUL1 as Marker for Pre-Eclampsia Progression

**DOI:** 10.21315/mjms2019.26.1.6

**Published:** 2019-02-28

**Authors:** Tjam Diana Samara, Isabella Kurnia Liem, Ani Retno Prijanti, Andrijono

**Affiliations:** 1 Doctoral Program in Biomedical Sciences, Faculty of Medicine, Universitas Indonesia, Jakarta, Indonesia; 2 Department of Anatomy, Faculty of Medicine, Trisakti University, Jakarta, Indonesia; 3 Department of Anatomy, Faculty of Medicine, Universitas Indonesia, Jakarta, Indonesia; 4 Department of Biochemistry and Molecular Biology, Faculty of Medicine, Universitas Indonesia, Jakarta, Indonesia; 5 Department of Obstetrics and Gynecology, Faculty of Medicine, Universitas Indonesia, Jakarta, Indonesia

**Keywords:** semaphorin 3B, cullin 1, serum, placenta, pre-eclampsia

## Abstract

**Background:**

An imbalance between pro- and anti-angiogenic factors contributes to impaired trophoblast invasion during pregnancy, leading to failure of uterine spiral artery remodeling, blood vessel ischemia, and pre-eclampsia (PE). Anti-angiogenic semaphorin 3B (SEMA3B) and pro-angiogenic cullin 1 (CUL1) are expressed in both the placenta and maternal blood. The present study investigated correlations between serum and placental SEMA3B as well as CUL1 levels in late-onset PE.

**Methods:**

This cross-sectional study included 50 patients with late-onset (≥ 32 weeks gestation) PE. Maternal serum was obtained before delivery, and placentas were obtained immediately after delivery. SEMA3B and CUL1 levels were evaluated by ELISA. Results were statistically analysed by Spearman correlation test, with a *P* < 0.05 considered statistically significant.

**Results:**

While elevated serum SEMA3B levels significantly correlated with increased placental SEMA3B levels in late-onset PE (*R* = 0.620, *P* = 0.000), alteration of serum CUL1 levels did not correlate with alteration of placental CUL1.

**Conclusion:**

Alteration of circulating maternal SEMA3B, but not CUL1, levels can potentially be used to monitor PE progression during pregnancy.

## Introduction

Pre-eclampsia (PE) is characterised by development of hypertension and proteinuria after 20 weeks of gestation or immediately after delivery (1). It affects approximately 2%–8% of all pregnancies and is one of the major causes of maternal and fetal morbidity and mortality (2). PE can be classified as early-or late-onset, each presenting with a different etiology (3). Stekkinger et al*.* classified early-onset PE as occurring before 32 weeks of gestation, and late-onset as occurring at or after 32 weeks of gestation (4). Unfortunately, the etiology and pathogenesis of PE still remain unknown. It has been proposed that PE is the result of an imbalance between anti- and pro-angiogenic factors during pregnancy. Normally, the levels of various anti-angiogenic factors elevate towards the end of pregnancy. However, PE is thought to involve an early increase in anti-angiogenic factors and/or excessive production of anti-angiogenic proteins, resulting in shallow endovascular invasion of cytotrophoblasts and pseudovasculogenesis failure (5). In turn, the spiral arteries do not dilate, vascular resistance increases, and patients develop hypertension and proteinuria (6).

Anti-angiogenic semaphorin 3B (SEMA3B) and pro-angiogenic cullin 1 (CUL1) are proteins expressed in both maternal blood and placental tissue known to play a functional role in pregnancy (7, 8). SEMA3B is a class 3 semaphorin/collapsin family member (9) containing a 749 highly conserved, NH_2_-terminal, semaphorin amino acids (10). SEMA3B has been identified as an inactive tumor suppressor gene found in lung cancer, ovarian cancer, hepatocellular carcinoma, and cholangiocarcinoma (11). Several studies have found increased SEMA3B levels in PE causes low trophoblast invasion. Zhou et al. (12) reported a significant increase of SEMA3B in PE cytotrophoblasts, while addition of SEMA3B to normal cytotrophoblasts inhibited invasion and recreated aspects of the cellular PE phenotype. Moreover, Wang et al*.* (13) revealed significant elevation of SEMA3B levels in maternal serum of PE subjects compared to controls. CUL1 is an essential component of the SKP1-CUL1-F-box protein E3 ubiquitin ligase complex (14) and plays a vital role in protein degradation and ubiquitination, mediating ubiquitination of proteins involved in cell cycle progression, signal transduction, and transcription (15). One study reported significantly lower CUL1 levels in human placental villi from PE patients compared to equivalent controls, indicating a role for CUL1 in trophoblast invasion (16).

So far, there have been no studies investigating both SEMA3B and CUL1 levels in both maternal serum and the placenta of the same PE subjects. Therefore, the present study investigated whether there is a correlation between maternal serum and placental levels of SEMA3B and CUL1 late-onset PE subjects. Therefore, the present study investigated whether there is a correlation between maternal serum and placental levels of SEMA3B late – onset PE subject. The results of this study will aid the study and identification of more effective biomarkers of PE.

## Materials and Methods

### Subjects

The present study had a cross-sectional design. Blood samples from 50 patients with late-onset PE (≥ 32 weeks of gestational age) were collected before delivery, and placental samples were obtained immediately after either cesarean section or vaginal delivery. Patients were recruited from Cipto Mangunkusumo Hospital and Budi Kemuliaan Hospital in Jakarta, Indonesia. All subjects were above 15 years of age and provided written informed consent prior to study inclusion. Subjects with diabetes mellitus and/or chronic kidney failure were excluded.

Late-onset PE was diagnosed and classified according to criteria recommended by the American College of Obstetrics and Gynecologists 2013 (1): new-onset hypertension developing after 20 weeks of gestation (systolic blood pressure ≥ 140 mmHg and/or diastolic blood pressure ≥ 90 mmHg), and proteinuria (≥ 300 mg in 24-h urine collection or +1 reading by dipstick) or without proteinuria, along with thrombocytopenia (< 100.000/μL), renal insufficiency (serum kreatinin > 1.1 mg/dL), liver dysfunction (transaminase level 2-times higher than normal), lung edema, cerebral disorder, or visual impairment.

### Measurement of Serum SEMA3B and CUL1 Levels in PE Patients

Blood (5 mL) was collected in vacutainer tube without an anti-coagulant from patients less than 24 h before delivery and then centrifuged at 3500 rpm for 10 min to clarify serum. Serum was collected and stored at −80 °C until assay use. Serum SEMA3B and CUL1 concentrations were determined with commercially purchased enzyme-linked immunosorbent assay kits (MyBiosource MBS2020622 and MBS921353, respectively).

### Measurement of Placental SEMA3B and CUL1 Levels in PE Patients

Placental tissue samples (0.5 cm × 0.5 cm × 0.5 cm) were obtained immediately after either vaginal delivery or cesarean section. Samples (approximately 100 mg) were washed in phosphate-buffered saline solution and then homogenised in 1 mL of phosphate-buffered saline. Placental homogenates were stored at −80 °C until assay use. Placental SEMA3B and CUL1 concentrations were determined with commercially purchased enzyme-linked immunosorbent assay kits (MyBiosource MBS2020622 and MBS921353, respectively, San Diego, CA, USA).

### Statistical Analysis

Data normality was tested with the Kolmogorov-Sminorv test, and the Spearman correlation test (non-parametric) was used on non-normal data to determine any correlations between serum and placental SEMA3B levels as well as CUL1 levels in late-onset PE patients. The data were analysed using the Statistical Analysis System, and a *P* < 0.05 was considered statistically significant.

## Results

Patient characteristics are presented in Table 1. The mean age of subjects was 32.22 years-old, with a mean gestational age of 36.46 weeks. The lowest and highest systolic blood pressures were 110 mmHg and 210 mmHg, respectively (mean, 157.96 mmHg), and the lowest and highest diastolic blood pressures were 70 mmHg and 140 mmHg, respectively (mean, 101.22 mmHg). Proteinuria was evaluated by qualitative measurement, with value undetectable until +4.

Mean levels of serum and placental SEMA3B were 0.253 and 1.912 ng/mL, respectively; mean levels of serum and placental CUL1 were 52.793 and 343.478 pg/mL, respectively (Table 2). Overall, SEMA3B and CUL1 levels in placental homogenates were approximately 7.5- and 6.5-times higher than those in serum, respectively (Figure 1). A significantly positive correlation was found between serum and placental homogenate SEMA3B levels in late-onset PE patients (R = 0.620, *P* = 0.000, Figure 2), suggesting an increment in serum SEMA3B may indicate increased placental SEMA3B prior to delivery. In contrast, there was no significant correlation found between serum and placental CUL1 levels (*R* = −0.095, *P* = 0.511, Figure 3).

## Discussion

To date, there have been no studies regarding correlations between the levels of serum and placental angiogenic factors, such as SEMA3B and CUL1, in late-onset PE. In a study of placental villous cytotrophoblasts from PE, preterm birth, and normal pregnancy patients at 23–39 weeks of gestation, Zhou et al. (12) reported that SEMA3B levels were highest in cytotrophoblasts and elevated in PE. They found that the autocrine action of SEMA3B plays a role in cytotrophoblast phenotypic changes, including impaired differentiation, signaling, and invasion, which are a primary problem in PE. SEMA3B was also shown to downregulate vascular endothelial growth factor (VEGF) signaling through phosphatidylinositol-3-kinase/AKT and glycogen synthase kinase 3 pathways, thereby controlling cytotrophoblast invasion by inducing apoptosis (12). Furthermore, a study of serum SEMA3B in 36 patients with PE compared to 36 normal pregnancies in the third semester by Wang et al. (13) found a significant increase in serum SEMA3B levels in PE compared to controls. They also reported that at 16–20 weeks of gestation, serum SEMA3B were significantly higher in those who eventually developed into PE compared to women with normal pregnancy.

Placental hypoxia is a known characteristic of PE (18) and may contribute to increased SEMA3B levels in placental explants. Wang et al. (13) reported that serum SEMA3B levels were elevated in the hypoxic placenta. On the other hand, Kaitu’u-Lino et al. (17) demonstrated that 48-h exposure of mature trophoblasts or placental explants to hypoxia significantly downregulated SEMA3B mRNA levels, but elevated SEMA3B protein. However, they did not find significant changes in SEMA3B mRNA expression or levels in the placenta from patients with severe early-onset PE (17). In the present study, however, serum and placental levels of two angiogenic factors in late-onset PE patients were compared and revealed increases in both serum and placental SEMA3B levels, with a much higher increment in the placenta. Moreover, these elevations showed a significant positive correlation, suggesting that anti-angiogenic SEMA3 can be used as a marker for detection of PE progression.

Meanwhile, only one previous study was found to have investigated the correlation between pro-angiogenic CUL1 and PE. In that study, CUL1 levels were found to be significantly decreased during syncytialisation in primary human placental cytotrophoblasts and significantly lower in the PE placental villous versus control (16). Their study also reported that CUL1 might play a role in the invasive ability of trophoblasts (16). In contrast, the current study did not find a correlation between the changes of serum and placental CUL1 levels in late-onset PE patients. These results align with a theory proposed by Bdolah et al. (5) in which decreased pro-angiogenic levels are not considered to be a cause of PE development. However, their theory does state that changes in anti-angiogenic protein production (e.g., gestationally early or excessive) due to other in vivo conditions (e.g., hypoxia) may lead to an imbalance of angiogenic factors, which is a known cause of PE development. Nonethless, further research into the role of pro-angiogenic CUL1 in PE is still necessary to better understand the molecular bass of this pathological process.

Initial studies on an imbalance of angiogenic factors in PE revealed increased soluble fms-like tyrosine kinase 1 (sFlt-1) levels in the circulation accompanied by decreases in both free circulating placental growth factor (PlGF) and VEGF (5, 19). Within 40 h after delivery, however, sFlt-1 levels began to decrease in PE patients. The elevation of sFlt-1 was suggested to be an anti-angiogenic event leading to endothelium dysfunction and clinical PE syndrome. Increased sFlt-1 expression in the placenta of PE patients accompanied by an increase in maternal circulating sFlt-1 (or vice versa) may suggest clinical onset of the disease and even be associated with its severity (19, 20). The role of SEMA3B as anti-angiogenic factor is similar to that of sFlt-1 via downregulation of VEGF (12). Taken together with the current results, this information suggests that maternal serum can be used to track changes in placental SEMA3B and sFlt-1 but not CUL1 in order to effectively monitor progression of PE.

There were some limitations to the present study. In particular, serum and placental SEMA3B and CUL1 levels from early-onset PE (< 32 weeks of gestation) and normal pregnancy patients of matched gestational age were not examined for comparison.

## Conclusion

The strong positive correlation between increased maternal serum and placental levels of anti-angiogenic SEMA3B, but not pro-angiogenic CUL1, in late-onset PE can potentially be used to monitor disease progression. However, further research regarding the role(s) of these factors, especially CUL1, in PE development and progression are necessary to confirm this conlcusion and better understand the molecluar mechanisms involved.

## Figures and Tables

**Figure 1:** Serum and placental SEMA3B and CUL1 levels in late-onset PE. Mean placental SEMA3B levels were approximately 7.5-times higher than those in maternal serum, while mean placental CUL1 levels were approximately 6.5-times higher

**Figure 2:** Correlation between serum and placental SEMA3B levels in late-onset PE. Spearman correlation testing (non-parametric) revealed a significantly positive correlation between serum and placental SEMA3B levels. *R* = 0.620; *P = 0.000

**Figure 3:** Correlation between serum and placental CUL1 levels in late-onset PE. Spearman correlation testing (non-parametric) did not indicate a significant correlation in CUL1 levels. *R* = −0.095; *P* = 0.511.

**Table 1:** Characteristics of late-onset pre-eclampsia subjects

Variable	*N*	Minimum	Maximum	Mean	SD
Maternal age (years)	50	20	44	32.22	5.563
Gestational age (weeks)	50	32	41	36.46	2.375
Systolic pressure (mmHg)	49	110	210	157.96	24.064
Diastolic pressure (mmHg)	49	70	140	101.22	12.185
Urine protein value (qualitative)	37	0	+4	+1.59	0.865

SD = standard deviation

**Table 2:** Serum and placental angiogenic factor levels in late-onset pre-eclampsia

Variable	*N*	Minimum	Maximum	Mean	SD
Serum SEMA3B (ng/mL)	50	0.790	0.625	0.253	0.153
Placental SEMA3B (ng/mL)	50	0.158	7.003	1.912	1.437
Serum CUL1 (pg/mL)	50	20.484	220.289	52.793	33.997
Placental CUL1 (pg/mL)	50	28.215	752.754	342.478	198.391

SD = standard deviation; SEMA3B = semaphorin 3B; CUL1 = cullin 1
